The article "Arabic Validity of the (CARE) Measure for Improving Medical and Mental Health Services" was retracted in 2023. Reasons: signs of a paper mill; suspected computer-generated content; unreliable results or conclusions; concerns about the data.

# Arabic Validity of the (CARE) Measure for Improving Medical and Mental Health Services

**DOI:** 10.1155/2022/6530019

**Published:** 2022-04-18

**Authors:** Abdelaziz Elfaki, Amani M AlQarni, Amal A. AlGhamdi, Malak A. AlShammari, Farheen Nasir, Rana Alabdulqader

**Affiliations:** ^1^Department of Psychiatry, College of Medicine, Imam Abdurrahman Bin Faisal University, Dammam, Saudi Arabia; ^2^Department of Family and Community Medicine, College of Medicine, Imam Abdurrahman Bin Faisal University, Dammam, Saudi Arabia; ^3^Department of Basic Science, King Saud Bin Abdulaziz University for Health Science, AlAhsa, Saudi Arabia; ^4^Medical Intern, King Fahd Hospital of the University, AlKhobar, Saudi Arabia

## Abstract

**Results:**

The majority of the item's responses showed high level of satisfaction. The coronach alpha of our study that examines the Arabic version of the CARE measurement tool 10 items was 0.96 showing an excellent internal consistency. The Kaiser-Meyer-Olkin measure was 0.96 indicating the adequacy of the data for factor analysis and the Bartlett test of sphericity shows (x^2^(45) = 8743.126, *p* < 0.001) indicating the adequacy of the correlation matrix for analysis.

**Conclusion:**

The Arabic version of CARE Measure seems to be consistent and reliable in the primary health care setting.

## 1. Introduction

Scientifically physician empathy is considered as an important component of consultations in primary health care and is crucial to the physician patient relationship. Physician empathy is defined clinically as the ‘‘socio-emotional competence of a physician to be able to understand the patient's situation, perspective and feelings, to communicate that understanding and check its accuracy, and to act on that understanding with the patient in a helpful (therapeutic) way” [1]. Patient perceptions of physician empathy has significant relation with patients' satisfaction with their physicians and clinicians, interpersonal trust, and compliance with physicians' recommendations as well as an added benefit to physicians in improving their diagnostic accuracy [2, 3]. Being an empathetic treating clinician, enables patients to cope better with their chronic illnesses both on subjective and objective parameters like reduced anxiety, better quality of life and clinical performance [4].

Improving clinical empathy is of interest to medical educators and health care authorities; finding an effective and convenient self-rated tool to be rated by patients is crucial to allow patient centered measures [5].

Many measurement tools of clinical empathy have been developed e.g. the EUROPEP questionnaire [6]. However, none of the scales are specific to family medicine clinics and suitable to be self-rated by patients without the need to be administered by physicians [7]. The consultation and relational empathy measurement tool (CARE) is broadly used in its ENGLISH version, it provides a specific, reliable, and patient centered estimate of perceived family physicians' clinical empathy [8].

The article "Arabic Validity of the (CARE) Measure for Improving Medical and Mental Health Services" was retracted in 2023. Reasons: signs of a paper mill; suspected computer-generated content; unreliable results or conclusions; concerns about the data.

Mercer and Reynolds have developed the CARE scale. It includes a 10-item self-administered measure involving four major domains assessed by the patients themselves to report an accurate conception of their experience. These are emotional, concerned with the patient's own experience, ethical, cognitive, and behavioral domains [1].

The CARE tool has been evaluated several times in the literature to prove its psychometric appropriateness and has been applied successfully in many high quality published research [8–10].

This tool, as stated previously, has been widely used in its original English language. No attempt to translate it to Arabic and use it has ever been made before. In our study, we aimed at examining the internal consistency and construct of the Arabic translated version of the CARE measurement tool.

## 2. Study Approval and Data Collection Methods

This is a cross sectional study that was done on 1245 patients of Imam Abdurrhman bin Faisal University's family medicine polyclinics for the period of June first, 2021–July first, 2021.

All patients during the data collection period were approached by our data collectors. The consenters then asked to fill up an anonymous noncompulsory self-administered electronic survey. The exclusion criteria was non-Arabic speakers and age less than 18 years old.

The research project was approved by the Ethics council at Imam Abdurrhman bin Faisal University (IAU), it complied with the policies and procedures of the institutional review board at IAU and granted approval with an IRB Number (IRB-2020-01-402).

## 3. The CARE Measure Description

The consultation and relational empathy (CARE) measurement tool was developed by Dr Stewart Mercer and colleagues to predict patient's perception of his/her physician's empathy.

It is a 10-item, with a 5-point Likert scale ranging from excellent [5] to poor [1] for each item. Up to two ‘Not Applicable' responses or missing values are allowed, and will be replaced with the remaining items' average score. Responses exceeding two ‘Not Applicable' responses or missing values are discarded from the analysis [8].

## 4. Translation

The (CARE) measure is originally in English language, and the English version was translated and back translated into Arabic by two independent professional translators. These versions were then discussed by a three bilingual consultant clinical psychologist. Pilot study was done on 32 patients to evaluate the understanding of the study participants to the language of the questionnaire, further amendments were done before the final version was released to be used for the actual study.

The article "Arabic Validity of the (CARE) Measure for Improving Medical and Mental Health Services" was retracted in 2023. Reasons: signs of a paper mill; suspected computer-generated content; unreliable results or conclusions; concerns about the data.

## 5. Analysis

The analysis was done using STATA software version 17. For the EFA and CFA the data set was randomly separated into two equal samples as the EFA was run on the first subsample whilst the CFA was run on the second one.

### 5.1. Exploratory Factor Analysis

Before running the EFA the data was examined for suitability of analysis using Kaiser–Meyer–Olkin measure and Bartlett test of sphericity. The estimation method of EFA was done using principal factor analysis and no rotation was administered. For choosing the factor number we depended on the retained Kaiser's criterion of Eigenvalue (>1) and scree plot. The significant factor loading was set to be > 0.3.

### 5.2. Confirmatory Factor Analysis

Maximum likelihood ratio estimation was chosen as the estimation method of the CFA. The root mean squared error of approximation (RMSEA; RMSEA<0.05), Tucker-Lewis index (TLI; TLI>0.95), comparative fit index (CFI; CFI>0.95), and the chi-square test (*p* < 0.05) were chosen to evaluate the model fit. Path modification was considered, based on the Lagrange test results.

## 6. Results

The total number of involved participants *n* = 1245. There was a wide variation amongst participants as the mean age of the study participants was 32.39 (SD = 13.89; min. = 18; max. = 85) and most of them were in their 1920s (*n* = 503, 40.37%). Male participants (*n* = 713, 57.27%) were more than female participants and majority of this study participants were Saudis (*n* = 1046, 84.02%). In addition, large number of participants were having college degree or higher (*n* = 901, 72.37%); however, many of them were unemployed (*n* = 772, 62.01%) as 93% (*n* = 718) of them were housewives **(**Table 1).

As seen in (Table 2), the majority of the item's responses showed high level of satisfaction as “letting you telling your story” item had the highest level of satisfaction (*n* = 934, 75%) chose “excellent” as their response. On the other side, the item “making plan action with you” had the lowest satisfaction as around *n* = 33, 2.54% reported “fair” or “poor” responses.

The coronach alpha of the of the CARE Measure tool 10 items was 0.96 showing an excellent internal consistency. The Kaiser-Meyer-Olkin measure was 0.96 indicating the adequacy of the data for factor analysis and the Bartlett test of sphericity shows (x^2^(45) = 8743.126, *p* < 0.001) indicating the adequacy of the correlation matrix for analysis.  Table 3 shows the polychoric correlation matrix summary that shows a good correlation and a common variance between the 10 items. The number of factors that were as guided by Kaiser's criterion and the scree plot (Figure 1) was one factor. The factor loading retained from the EFA is summarized in (Table 4) and it is seen there that the factor loading that is (>0.3) was only seen in relation to factor 1.

The article "Arabic Validity of the (CARE) Measure for Improving Medical and Mental Health Services" was retracted in 2023. Reasons: signs of a paper mill; suspected computer-generated content; unreliable results or conclusions; concerns about the data.

The CFA that was run on the other half of the data to confirm the EFA analysis results showed an excellent model fitting statistics as following; x^2^(35) = 359.464, *p* < 0.001; REMSEA = 0.122 (CI = 0.111 to 0.134); CFI = 0.959; TLI = 0.948 which indicate the suitability of this run latent model. The estimation results of the CFA are summarized in Figure 2.

In summary, the Arabic translated version of CARE Measurement tool showed an excellent internal consistency and its internal construct showed only one latent factor that was explained by all the 10 items with an excellent CFA fitting model statistics.

Table 2 summarises the distribution of the participants responses to the 10 items of the CARE measurement tool (*n* = 124).

Extraction method = principal factor analysis; rotation method = unrotated, loading larger than 0.4 is in bold.

## 7. Discussion

We translated and validated in this study the original English version of the CARE Measurement tool into Arabic language in a primary health care facility (PHC) of a university hospital in Eastern province, Saudi Arabia. Table 1 is for the demographic information showing total 1245 participants were involved which included both patients 75.42% and caregivers 24.58%. The mean age range of the participants was 32.39; male female ratio was 713 : 532. 84.02% of the participants were Saudi nationals while 15.98% belonged to other nationalities.72.37% of the participants had college or higher-level degrees but 62.01% were unemployed. In Table 2 all the 10 items of the CARE measure show high level of satisfactory responses by the participants. A study on the check of the validity and reliability of the CARE measure showed high satisfaction responses by the patients where it was not affected by the demographic differences [11].

In the Arabic CARE Measure, the number of “not applicable” was very low in almost all the items. The lowest was 0% in the third item, stated as “really listening” and the highest was 2.01% in item seven, stated as “being positive”. For the rest of the three items, namely no. 8, 9 and 10, “not applicable” was selected 1.77% of the time. Items 8, 9, and 10 were stated as “explaining things clearly”, “helping you to take control” and “making a plan of action with you”, respectively and all were based on the cognitive and behavioral aspects of empathy. One reason for this can be the concept of shared responsibility with the patients rather than sole responsibility of the physicians as indicated in the Swedish version CARE [12] measure Moreover the number of responses in the poor category was very low as majority had responded in the very good and excellent categories.

The article "Arabic Validity of the (CARE) Measure for Improving Medical and Mental Health Services" was retracted in 2023. Reasons: signs of a paper mill; suspected computer-generated content; unreliable results or conclusions; concerns about the data.

The two statistical techniques which were utilized to measure the validity and reliability of the Arabic version of (CARE) measurement tool were Exploratory Factor Analysis (EFA) and Confirmatory Factor Analysis (CFA). EFA which was done on the first half of the sample and as summarized in Tables 2 and 4 shows that the factor loading (>0.3) was only seen in relation to factor 1.

Cronbach's alpha with a score of 0.96 showed an excellent internal consistency and CFA which was run on the second half of the sample both have confirmed internal structure consistency of the Arabic CARE Measurement tool and consensus with the original, Chinese, and Japanese versions of the CARE Measure [13, 14]. [1–3] As a result, external and internal validity of the Arabic CARE Measurement tool is sustained.

Table 2 shows polychoric correlation matrix of all the 10 items with each other. All the items show strong above average correlation except for item no. 3 whose correlation with the rest of the 9 items lies in the average range minimum *r* = 0.69 to maximum *r* = 0.73.

One of the study strength points that it was conducted on a large sample, and there was no missing data as all the 1245 responses were available for all the 10 items of the scale. Similar findings were discovered with extremely low “missing values” and “not applicable” data in a research on the patients of secondary care in Scotland [11]. This study indicated CARE measure to be considered as highly relevant with internal and structural reliability plus face and concurrent validity.

In a study CARE measure was also used for validity and reliability check on primary care nurses and the results showed that it has high face and construct validity and internal reliability for the nurses working in the primary care of the patients [15]. Another study done on the rehabilitation patients in the Southern England showed that CARE fulfilled the strict standards for internal construct validity [16].

## 8. Limitations

The study was conducted in a single primary health care in eastern province, Saudi Arabia, and is limited to university employees, hospital employees, students, and their families. Therefore, conducting the same study on different primary health care centers, different specialized clinics in different provinces of Saudi Arabia will aid in improving overall patients' satisfaction.

The article "Arabic Validity of the (CARE) Measure for Improving Medical and Mental Health Services" was retracted in 2023. Reasons: signs of a paper mill; suspected computer-generated content; unreliable results or conclusions; concerns about the data.

## 9. Recommendations

It is recommended to develop a CARE measure to be used for the virtual clinics, as after the Pandemic use of the virtual clinic facilities have also become quite common.

## 10. Conclusion

The original CARE Measurement measure was translated and validated in Arabic, and the study was done in a primary health care context. The Arabic format of the CARE Measurement instrument appears to be consistent, trustworthy, and valid in the primary health care context; nevertheless, more study in different locations across the nation is required.

## Figures and Tables

**Figure 1:** scree plot for exploratory factor analysis that was done on the first half of the sample (*n* = 623).

**Figure 2:** Confirmatory factor analysis; estimation method ML that was run on half of the participants (*n* = 622). The latent variable is represented with an oval shape whilst each item is represented with a square. The small circles represent the estimation error whilst the arrow represents the regression line.

**Table 1:** Characteristics of study participants (*n* = 1245).

	*N* = 1245	%
Age groups		
<20 years	69	5.54
20–29 years	503	40.37
30–39 years	301	24.16
40–49 years	168	13.48
50–59 years	132	10.59
60–69 years	57	4.57
70–79 years	12	0.96
≥80 years	4	0.32
Gender		
Female	532	42.73
Male	713	57.27
Nationality		
Saudi	1046	84.02
Non-Saudi	199	15.98
Partnership		
Without partner	632	50.76
With partner	613	49.24
Educational level		
High school and lower	344	27.63
College and higher	901	72.37
Employment status		
Employed	473	37.99
Nonemployed	772	62.01
Patient or patient caregiver		
Patient	939	75.42
Caregiver	306	24.58

**Table 2:** The distribution of participant's responses (*n* = 1245) of CARE questionnaire questions.

	Responses											
	Poor		Fair		Good		Very good		Excellent		Not applicable	
Items	n	%	n	%	n	%	n	%	n	%	n	%
1. Making you feel at ease	5	0.40	17	1.37	85	6.83	214	17.19	912	73.25	12	0.96
2. Letting you tell your “story”	4	0.32	13	1.04	80	6.43	195	15.66	934	75.02	19	1.53
3. Really listening	6	0.48	18	1.45	79	6.35	239	19.20	903	72.53	00	0.00
4. Being interested in you as a whole person	8	0.64	15	1.20	84	6.75	216	17.35	905	72.69	17	1.37
5. Fully understanding your concerns	9	0.72	23	1.85	89	7.15	199	15.98	901	72.37	24	1.93
6. Showing care and compassion	6	0.48	19	1.53	83	6.67	208	16.71	909	73.01	20	1.61
7. Being positive	6	0.48	8	0.64	94	7.55	205	16.47	907	72.85	25	2.01
8. Explaining things clearly	8	0.64	16	1.29	93	7.47	212	17.03	894	71.81	22	1.77
9. Helping you to take control	8	0.64	19	1.53	87	6.99	214	17.19	895	71.89	22	1.77
10. Making a plan of action with you	9	0.72	22	1.77	90	7.23	204	16.39	898	72.13	22	1.77

The article "Arabic Validity of the (CARE) Measure for Improving Medical and Mental Health Services" was retracted in 2023. Reasons: signs of a paper mill; suspected computer-generated content; unreliable results or conclusions; concerns about the data.

**Table 3:** The polychoric correlation matrix of the 10 items of CARE measurement tool (*n* = 1245).

		1	2	3	4	5	6	7	8	9	10
1	Making you feel at ease	1.00									
2	Letting you tell your “story”	0.92	1.00								
3	Really listening	0.74	0.70	1.00							
4	Being interested in you as a whole person	0.88	0.93	0.74	1.00						
5	Fully understanding your concerns	0.87	0.93	0.74	0.94	1.00					
6	Showing care and compassion	0.86	0.90	0.72	0.94	0.94	1.00				
7	Being positive	0.90	0.93	0.69	0.96	0.94	0.96	1.00			
8	Explaining things clearly	0.85	0.91	0.70	0.91	0.92	0.95	0.94	1.00		
9	Helping you to take control	0.87	0.89	0.69	0.91	0.90	0.94	0.95	0.95	1.00	
10	Making a plan of action with you	0.88	0.90	0.73	0.91	0.90	0.92	0.93	0.92	0.95	1

**Table 4:** The factor loadings of the 10 items of the CARE measurement tool that was gain from the exploratory factor analysis that was run on the first half of the sample (*n* = 623).

Number	Items	Factor 1	Factor 2	Factor 3	Uniqueness
1	Making you feel at ease.	**0.92**	0.18	0.02	0.12
2	Letting you tell your “story”	**0.95**	0.09	-0.10	0.07
3	Really listening	**0.75**	0.23	0.13	0.37
4	Being interested in you as a whole person	**0.97**	0.04	-0.09	0.06
5	Fully understanding your concerns	**0.96**	0.05	-0.08	0.07
6	Showing care and compassion	**0.97**	-0.10	-0.03	0.05
7	Being positive	**0.98**	-0.09	-0.09	0.03
8	Explaining things clearly	**0.96**	-0.14	0.03	0.06
9	Helping you to take control	**0.96**	-0.16	0.11	0.04
10	Making a plan of action with you	**0.95**	-0.04	0.14	0.07

## Data Availability

The data used to support the findings of this study are included within the article.
